The article "Analysis of the Influence of Rural Family Education Environment on School-Age Children's Social Behavior and Patterns" was retracted in 2023. Reasons: unreliable results or conclusions; concerns about the data; concerns about the results or conclusions; concerns about the peer review.

# Analysis of the Influence of Rural Family Education Environment on School-Age Children's Social Behavior and Patterns

**DOI:** 10.1155/2022/3594462

**Published:** 2022-08-08

**Authors:** Wenwen Yao, Ying Zhen, Yu Zhang

**Affiliations:** School of Educational Science, Mudanjiang Normal University, Mudanjiang Heilongjiang, 157011, China

## Abstract

Family education will have an important impact on children's body and psychology. It is different from social education and school education. It is mainly based on parents' words and deeds. Children enhance their life experience through the family's living atmosphere. Restricted by geographical conditions and economic level, family education is not given enough attention, and children's social behavior is more prone to problems. Therefore, rural primary more needed to pay attention to the impact of family education on children and promote the healthy development of children's physical health. Children's social disorder behavior is currently the most common phenomenon that hinders the normal development of children's interpersonal relationships in the physical and mental development of children in my country. This problem is not only reflected in the psychology of children with social disabilities, but also in normal children and children with social disabilities in daily social interactions. In the current product design market, a single product cannot comprehensively solve the practical problems encountered by children with social disabilities. Therefore, it is necessary to explore the possibility of experience design with multidimensional perspectives and multidisciplinary integration. This paper analyzes the current situation of children's social behavior in a rural family education environment and expounds the problems existing in rural family education and the impact of rural family education on children's social behavior. To provide a reference for improving children's social behavior in my country.

## 1. Introduction

Children's education refers to the training and training of moral education, intellectual education, and physical education. Children's education is the foundation of education. As General Secretary Xi Jinping said, “The buttons of life should be buttoned right from the beginning. If the first button is buttoned wrongly, the rest will be buttoned wrongly.” He is in Haidian National Primary School. General secretary of the Communist Party of China (CPC) Central Committee Xi Jinping said on the Party's 18th National Congress, “As long as you follow the right path from childhood, learn a little, practice a little, and strive to be the best of me, in my best aspect, life will usher in sunshine all the way.” It is clearly pointed out that education is the cornerstone of national rejuvenation and social progress, education is the foundation of national prosperity, education is strong, the country is strong, and ideological and political education is the foundation of life after all [1]. On September 10, 2016, the General Secretary emphasized that basic education is a social undertaking and requires close cooperation between schools, families, and society [2]. In short, it is necessary to always run through the people-oriented educational concept, combine the actual situation of family, school, and society, and earnestly in practice, do a good job in primary education, and integrate family ideological and moral education into the development of students' ideological and moral behavior [3].

The article "Analysis of the Influence of Rural Family Education Environment on School-Age Children's Social Behavior and Patterns" was retracted in 2023. Reasons: unreliable results or conclusions; concerns about the data; concerns about the results or conclusions; concerns about the peer review.

In total, 0–3 years old is a critical period of child development and the foundation of human development. Preparing for early childhood development is of great significance to the improvement of human capital in the future. Including family early education, exercise children's physical fitness, intelligence, psychological ability, improve children's sense of security, willpower, and sense of goal. Improving human capital from the source can provide a long-term driving force for the stable development of the economy. The good development of social emotions in early childhood lays the foundation for later entry into the social environment [4]. There is overlap in developmental domains and behavioral processes between social competence and emotional competence, the set of behaviors that enable someone to establish and engage in positive interactions with peers, siblings, parents, and other adults [5]. Many scholars at home and abroad have studied the current situation and influencing factors of children's social-emotional development. Children in urban areas, and there is less literature on children in rural areas [6].

The decrease in the number of peers among family members has led to preschool children being unwilling and not used to communicating with others, and also prematurely bearing family and social pressures [7]. The root causes of mental stress in only child children are motivational conflict, socioeconomic status, educational institution status, and psychological trauma. Excessive care and spoiling also prevent some only children from developing their cognitive abilities in a healthy way [8]. The year-on-year increase in the number of children with autism is a good example. Although the advancement of technology has enriched the way of entertainment for preschool children, for preschool children, electronic devices full of technological sense are constantly tempting children [9]. They spend most of their time playing video games instead of participating. In outdoor activities, there is little contact with the external environment, so he has very little understanding of himself and others and even social knowledge of society [10]. As a result, school-age children have social behavior phobia, and in different places, the degree of social phobia is different, as shown in Figure 1.

The article "Analysis of the Influence of Rural Family Education Environment on School-Age Children's Social Behavior and Patterns" was retracted in 2023. Reasons: unreliable results or conclusions; concerns about the data; concerns about the results or conclusions; concerns about the peer review.

## 2. Theoretical Research

### 2.1. Overview of Rural Family Education Theory

The concept of “rural” in this article is mainly defined from the aspects of population, production activities, and economic development level, which refers to residential settlements that are mainly engaged in agricultural production activities compared with cities, and the population is relatively scattered, and there is a significant gap with the urban economic level. Family education generally refers to the activities that parents carry out for their children's study and life. Sun Junsan divides family education into broad and narrow senses in his book “Family Pedagogy Fundamentals” [11]. In a broad sense, family education is “1. A kind of education implemented by family members; Human ideology and morality, and activities to develop human intelligence and physical strength are all education [12].” In a narrow sense, family education refers to “under a certain family cultural background, the parents or other elders impose certain influences on minor children or juveniles. Educational influence activities that help them socialize and form a sound personality, moral, intellectual, and physical development [13]”.

Children of different ages have different social behaviors, as shown in Table 1. Children in elementary school begin to learn knowledge and skills, and gradually form a sense of success and achievement through diligence, and their concentration is not strong, they are easily disturbed by the outside world, their willpower is relatively weak, and they may have low self-esteem in the face of failures and setbacks. Children at this stage have the most important relationship with their peers [14]. In terms of emotional expression, they are more exposed, unstable, and lasting [15]. If parents pay attention to and guide their children's education in a timely manner, it will help reduce this stage. The harm caused by the existential crisis can be reasonably resolved, these are indispensable factors for the child's later academic achievement and self-concept formation [16].

### 2.2. The Social Behavioral Implications of School-Age Children

The so-called social behavior refers to “the process in which a biological person as an individual grows into a social person and gradually adapts to social life [17]. Through this process, the social culture is accumulated and continued [18], the social structure is maintained and developed, and the person's personality is formed and perfected” [19]. The socialization of children has always been a key issue in sociology and sociology of education research. Studying the significance of children's socialization can help improve awareness of children's psychological development. In the early days of human society, education was essentially synonymous with socialization. Later, due to the development of social productive forces, in the process of conquering and transforming nature, people increasingly needed professional techniques and means, and the emergence of specialized educational institutions made education and socialization distinguishable [20]. It can be seen that education and socialization are closely related, and education is not completely equivalent to socialization, but family education is an important way to realize children's socialization, and socialization itself also depends on school education and family education.

The article "Analysis of the Influence of Rural Family Education Environment on School-Age Children's Social Behavior and Patterns" was retracted in 2023. Reasons: unreliable results or conclusions; concerns about the data; concerns about the results or conclusions; concerns about the peer review.

Sociology of education research on children's socialization is very meaningful. For children's individual socialization, it is “a necessary precondition for individuals to adapt to society, participate in social life, and survive independently in the social environment”. In the process of growing from “natural person” or “biological person” to “social person”, children must go through necessary social education. Only by mastering the laws and skills of social life can we survive in society; and the socialization of children cannot be completed at one time, and the changes in human society have caused great changes in society in terms of ideology, moral norms, and institutions, making it difficult for individuals to adapt to social changes. The process of socialization plays different roles, and it is of great significance to study the different characteristics of the two in children's socialization for how to better realize children's socialization.

### 2.3. Classification of Children's Social Disorder Behavior

In the definition of psychology, the concept of children's social disorder is explained in both broad and narrow senses. In the narrow sense, childhood social disorder is defined as a child's emotional disorder, which is within the scope of psychology. It is listed in the “American Diagnostic and Statistical Manual of Mental Disorders, Fourth Edition”, Social Psychological Disorder and Selective Mutism, Children's Separation Anxiety Disorder, Children's Social Anxiety Disorder, Social Dysfunction, etc. The broad concept includes not only mood disorders specific to childhood, but also various types of adult neuroses that appear in childhood, such as phobic neurosis, anxiety neurosis, obsessive-compulsive neurosis, depression, and neurosis and hysteria. From a theoretical point of view, family education has always been an active topic in the academic community, and it is also a hot topic for experts and scholars to study.

The article "Analysis of the Influence of Rural Family Education Environment on School-Age Children's Social Behavior and Patterns" was retracted in 2023. Reasons: unreliable results or conclusions; concerns about the data; concerns about the results or conclusions; concerns about the peer review.

## 3. Analysis of Social Behavior Problems in School-Age Children

Under the pressure of fast-paced development and severe competition in today's society, mental health problems have attracted the attention of the majority of society. The negative effects are huge. Social terror refers to the fear of interpersonal communication. Patients often try to avoid the social environment, and the symptoms of direct interpersonal contact appear in the process of tension and anxiety. Previous studies have shown that the proportion of children and adolescents with social phobia is much higher than that of other age groups. According to conservative estimates, there are at least 30 million to 50 million preschool children in my country with behavioral problems. And children's fear objects are also different in different periods, as shown in Figure 2. The family is the child's first school, and the parents are the child's first teacher.

### 3.1. Social Phobia in Children

Children's social phobia is a common childhood emotional disorder, which refers to children's persistent fear, anxiety, and avoidance behaviors in unfamiliar environments or strangers, but social relations are good when they are with family members or in familiar environments. The behavior of social anxiety will continuously affect the development of children's physical and mental health, such as avoiding social interaction, reducing social exercise, declining learning ability, and lack of social ability, which will have many negative effects on the development of children throughout their lives. Not only that, if children's social phobia cannot be intervened and corrected in time, it will lead to social estrangement in the long run, social deviant behavior will occur, and it is not surprising that it will turn into a morbid state. The vicious circle of children's social phobia is shown in Figure 3. Various psychological or behavioral problems that arise in adulthood also largely reflect the problems and deficiencies that existed in childhood. Therefore, find the root of the problem, use the theoretical knowledge and methods of social work to deeply analyze the problem of children's social fear behavior and its causes, and provide professional services to help children eliminate social barriers and restore social skills, so as to provide social support for adolescents and children. Early intervention for fear provides direction.

The article "Analysis of the Influence of Rural Family Education Environment on School-Age Children's Social Behavior and Patterns" was retracted in 2023. Reasons: unreliable results or conclusions; concerns about the data; concerns about the results or conclusions; concerns about the peer review.

### 3.2. Assessment Methods for Children's Social Phobia

Regarding the evaluation criteria of social phobia, researchers generally make a comprehensive evaluation of the patient's internal thinking, feeling, and external behavior from the perspectives of cognition, behavior, and body. The social fear and anxiety scale developed by Turner are shown in Table 2 and the social anxiety scale and social interaction anxiety scale are developed by Mattick. Social Function Assessment Scale SPRS, published in 1998, is the latest scale for assessing external behavior in patients with social phobia. The scale evaluates the behavioral performance of the subjects from five aspects.

The assessment of social phobia in the United States is largely based on the Diagnostic Statistical Manual of Mental Disorders, 4^th^ revised edition (DSM-IV). It is very difficult to diagnose children's social anxiety. For example, children's social anxiety behavior is regarded as “shy and introverted” by adults. These can all lead to false diagnoses of the child's condition. Some scholars believe that the RICE social ladder can be used for evaluation, as shown in Figure 4. The RICE social ladder evaluation system is based on more than 10 million pieces of project data, combined with AI artificial intelligence technology, and developed for the social characteristics of Chinese children, which can effectively evaluate children's social barriers. The research on social phobia in China started late, and the assessment tools for social phobia are relatively lacking. Current research mainly uses self-reported or other-rated psychological scales to reflect the severity and efficacy of patients' symptoms.

### 3.3. Research on the Formation Factors of Children's Social Phobia

In the research on the causes of children's social anxiety, one of the more studied abroad is the parenting style, which is also considered to be a factor closely related to the development of social anxiety disorder. Parental upbringing characteristics such as overcontrol, lack of family warmth, rejection, and overprotection are all related to the causes of children's social anxiety. Low education level is also a factor in the formation of social fear. For example, individuals who have not received a college education have a significantly increased degree of social fear. Specifically as shown in Figure 5.

A study by Chartier and Walker found that some major negative life events experienced in childhood increase the risk of developing the disease in children. In the domestic research on the causes of children's social phobia, it is believed that there is no statistical difference in social phobia between males and females. Some psychological researchers believe that social phobia is influenced by psychological factors. Most studies also show that family factors are an important factor that cannot be ignored in the causes of children's social phobia. The company of parents to children can reduce the anxiety level of children. Improper parenting methods can easily make children anxious. The influence of family time with children on whether children have social barriers is shown in Figure 6.

The article "Analysis of the Influence of Rural Family Education Environment on School-Age Children's Social Behavior and Patterns" was retracted in 2023. Reasons: unreliable results or conclusions; concerns about the data; concerns about the results or conclusions; concerns about the peer review.

The family's surrounding environment has a profound impact on children's social ability and is an important factor affecting the incidence and prognosis of SPDC, as shown in Table 3. In particular, the parenting style of the mother is the most important. In the process of problem-solving, the more the mother controls and restricts, the higher the anxiety level of the children in the future. In addition, relationship aggression, physical aggression, and social anxiety in middle childhood peer aggression were significantly positively correlated.

## 4. Research on Countermeasures of Rural Family Education to Promote Social Behavior of School-Age Children

### 4.1. Build Good Family Relationships

In order to build a good relationship between children and parents, more communication is needed, especially in remote areas such as rural areas. At present, China is accelerating the construction of new rural areas, paying attention to farmers, rural areas, and agriculture. The accelerated development of the economy has brought great impetus to the development of rural areas. In this context, parents take the initiative to communicate with their children, which reflects their care and love for their children, but when children take the initiative to communicate with their parents, it shows that the children trust their parents more. In order to consolidate this relationship, parents must pay attention to communication skills. In the process of communication, a negotiated tone is often used. Children are very disgusted by parents adopting an imperative tone, especially when pointing out children's wrong ideological and moral behavior and bad behavior. Rebellious mentality: use a negotiating tone or a suggestive tone to communicate with your children. They will be willing to make corrections, be good to each other, and will not affect the development of the parent-child relationship.

### 4.2. Reshape the Concept of Family Education and Build a Learning-Oriented Family Education

Family education has a lifelong educational role in the family. Family education runs through the growth process of children, and it has a very important position in the entire education system. It is necessary to change from the low-level traditional family education concept focusing on childcare, and establish a modern family education concept. A good personality is a requirement, and finally a joint force of family education is formed, so that children can initially form.

The article "Analysis of the Influence of Rural Family Education Environment on School-Age Children's Social Behavior and Patterns" was retracted in 2023. Reasons: unreliable results or conclusions; concerns about the data; concerns about the results or conclusions; concerns about the peer review.

Self-awareness and social role awareness, with sound personality and good social norms, developed intelligence and a strong physique. To this end, it is necessary to start with building a learning-oriented family education, establish a correct concept of family life, carry out beneficial family life activities, adjust the family consumption structure according to the family's economic situation, and form a good parent-child relationship and harmonious family atmosphere. The basic literacy of family members maintains a good family learning environment and implements family education in an equal, democratic, and cordial atmosphere; parents must have a sense of modernization and have a scientific concept of parent-child and parenting, which is important for building a learning family and children. Socialization goes a long way.

### 4.3. Family Education Training for Parents

Without scientific family education, it is difficult for many teachers to communicate effectively with parents, and the school's parent education work will not be effective. First of all, parents must be made aware of the relationship between social changes and the family. In 1982, the state introduced family planning to encourage only one child to improve the quality of the population. Although this policy has controlled the population, it failed to ensure the quality of the population and caused serious problems. With the phenomenon of aging, it is obvious that children are the “jewel in the palm” of the family, and a large number of “incompetent children” have appeared, which have seriously hindered the country's economic development. Until 2016, when the “two-child policy” corresponding to family planning was fully implemented, a family of three gradually developed into a family of four. Social development followed the changes in the family structure, and the relationship and life among family members also changed. With the change, the function of family education has gradually improved.

Parents must first understand the characteristics of children's development at different stages and master the laws of children's psychological development, as well as their needs at different stages, and carry out family parenting education in a targeted manner. Second, communicate effectively with children, know how to communicate diligently, communicate in the way of treating “little adults”, and eliminate the formal level difference, such as squatting down to communicate with children, eliminating the spiritual level difference, communicating sincerely, increasing Intimacy and avoiding estrangement are the most important things. Finally, pay attention to children's moral behavior problems at all times, and deal with them in time and correct them. The quality of academic performance does not represent everything. If you have acquired correct moral theoretical standards in textbooks, if you do things in different ways in life, parents should make timely judgments, and deal with efficiently.

The article "Analysis of the Influence of Rural Family Education Environment on School-Age Children's Social Behavior and Patterns" was retracted in 2023. Reasons: unreliable results or conclusions; concerns about the data; concerns about the results or conclusions; concerns about the peer review.

### 4.4. Strengthen the Guidance of Family Education in Schools

First of all, it is necessary to strengthen the connection between home and school. There are many ways to combine parents and schools, such as parent education, parent visits, written communication, and family visits. Home visits are one of the means of combining school and family education. This is the responsibility of every teacher. Through home visits, teachers and parents can increase their understanding of children in different aspects. In the region, very few teachers have received training on visits. In the process of the home visit, how to start and how to understand through observation rather than inquiry is worth learning and discussion by teachers. For example, in family visits of single-parent families, children will be influenced by their fathers and mothers in which aspects, and whether they attach importance to the development of parent-child relationship. Some children are taken care of by their grandparents and spend too little time with their parents. Moreover, today's children rarely listen to the older generation. Parents will only occasionally reprimand children with behavioral problems and cannot solve and correct and so on. These are all issues that teachers need to pay attention to when making home visits.

From the perspective of schools, the traditional education model should also be innovated. The educational goals of the lower grades of basic education should be completely transformed from the single goal of systematic knowledge mastery, to establish the mastery of knowledge and the development of students' basic skills in life, and to form an educational philosophy of moral norms and values. This concept reforms the content of school education, innovates the teaching material system, pays attention to the content of basic social norms education, combines the traditional Chinese humanistic spirit with the basic requirements of modern society, improves children's humanistic quality, and enhances children's humanistic spirit. At this end, it is necessary to implement a variety of educational methods, focusing on the implementation of activity classes, and through games, to strengthen interaction in various forms such as social visits and discussions that are in line with children's individuality, enhance children's perceptual awareness, improve children's ability to distinguish right from wrong, and achieve education target.

The article "Analysis of the Influence of Rural Family Education Environment on School-Age Children's Social Behavior and Patterns" was retracted in 2023. Reasons: unreliable results or conclusions; concerns about the data; concerns about the results or conclusions; concerns about the peer review.

## 5. Conclusion

Children are the future and hope of the motherland. It is the responsibility of every parent to educate them to grow into talents. It is also a course for every parent to “learn by doing”. Family education is the most basic and most important part of education. The healthy growth of children is inseparable from the cultivation of the family. From ancient times to the present, China attaches great importance to family education, and the three migrations of Mengmu are a classic example, so many outstanding scholars have emerged in the field of family education. Therefore, every step in the right direction will be conducive to future growth. Parental education, as the leader of children's life, must not only play the role of escort, but also be an out-and-out instructor. Obviously, family education is the fundamental education for children's thinking and behavior learning. Through the research on rural family education and the theory of children's social disorder, this paper analyzes the causes of children's social disorder and related evaluation methods and puts forward corresponding countermeasures and suggestions by analyzing the impact of rural family education on children's social behavior. It has important reference significance for promoting children's mental health development and solving children's social barriers.

## Figures and Tables

**Figure 1:** Social fear scenarios for school-age children.

**Figure 2:** Fear objects of school-aged children at different times.

**Figure 3:** The vicious circle of children's social fear behavior.

**Figure 4:** RICE Social Ladder Review estimate.

**Figure 5:** The effect of parental education on the social behavior of school-age children.

**Figure 6:** The effect of family time spent with children on whether children have social barriers.

**Table 1:** Social behaviors of children at different ages.

Development tasks	Social environment	Coordinating behavior	Development history monument	Age
Adjust	Mainly parent-child relationship	Parents help babies regulate sleep, eating, distress, and arousal levels	Develops attention to the social world, increasing regulation of parent-infant interactions	0–3
Demonstration of social competence	Mainly parent-child relationship	Parent-led parent-infant coordination; more extended face-to-face communication; parents begin verbal communication with infants	Increased eye contact; display of a social smile; social language	2–3
Reciprocal swap	Parent-child relationship, close family relationship	Babies communicate back and forth with others	Infants are increasingly adapting to social responses	3–6
Baby's initiative	Parent-child relationship, close family relationship	Infants begin to play with others and increase direct mobility; infants groom others' behavior	Intentional and goal-directed - infants show a preference for certain activities and attract attention; enjoys games (e.g, peek-a-boo)	6–9
Occurrence and establishment of focused attachment	Parent-child relationship	Parents provide a foundation of safety: Infants feel comfortable with their parents and rely on their parents for protection during distress; infants explore their environment under parental protection	Stranger anxiety; separation anxiety; permanent presence of individuals (perceived presence of parents even in their absence); basic safety behaviors	7–18
The emergence of shared attention	Enlarged environment including parents, family members, peers, and guardians	Infants demonstrate awareness of others' perspectives; infants seek out other people's facial expressions to learn about new situations	Imitation learning; social referencing; exhibiting instrumental, purposeful responses	9–12
Confident and independent self-concept	Enlarged environment including parents, family members, peers, and guardians	Infants are self-aware; infants decide and choose their own goals and intentions apart from their parents	Mirrored self-perception; use of “no” and tantrums; increased autonomy; self-centered reasoning	18–24
Goal correction partnership	Enlarged environment including parents, family members, peers, and guardians	The child exhibits a new awareness when the caregiver's attention is separated from him or her; the communication between two autonomous but interdependent individuals is increasingly coordinated	Persistent primary relationships and permanent appearance of objects; behaviors that improve negotiating skills and coordinate other goals: Empathic behaviors	18–36
Build peer relationships	Siblings, peer relationships	Children engage in meaningful interactions with siblings and peers in playgroups, daycare settings, and other settings	Increased interest in other children; from loneliness to parallel play: play with peers, empathy, and concern for peers' distress	18–36

The article "Analysis of the Influence of Rural Family Education Environment on School-Age Children's Social Behavior and Patterns" was retracted in 2023. Reasons: unreliable results or conclusions; concerns about the data; concerns about the results or conclusions; concerns about the peer review.

**Table 2:** Social interaction anxiety scale.

Fear subjective scale measure (unit sub)				
0	25	50	75	100
Calm mood	Mild fear	Moderate fear	High fear	Extreme fear

**Table 3:** The influence of family surrounding environment on children's social behavior.

Are there social places	Frequency	Do preschool children have social impairments?		Total
	OK%	Yes	No	
Have a social place	Frequency	42	30	72
	OK%	58.3	41.7	100

No social place	Frequency	372	56	428
	OK%	86.9	13.1	100

Total	Frequency	414	86	500
	OK%	82.8	17.2	100

## Data Availability

The labeled dataset used to support the findings of this study is available from the corresponding author upon request.
